# Detection of Bone Metastases by ^68^Ga-DOTA-SSAs and ^18^F-FDG PET/CT: A Two-Center Head-to-Head Study of Gastroenteropancreatic Neuroendocrine Neoplasms

**DOI:** 10.1155/2022/1750132

**Published:** 2022-11-07

**Authors:** Rui Tian, Qing Xie, Fei Yu, Changzhi Du, Xiaochen Yao, Shiming Zang, Chuan Zhang, Pengjun Zhang, Guoqiang Shao, Zhi Yang, Feng Wang, Jiangyuan Yu

**Affiliations:** ^1^Department of Nuclear Medicine, Nanjing First Hospital, Nanjing Medical University, Nanjing 210006, China; ^2^Key Laboratory of Carcinogenesis and Translational Research (Ministry of Education/Beijing), Key Laboratory for Research and Evaluation of Radiopharmaceuticals (National Medical Products Administration), Department of Nuclear Medicine, Peking University Cancer Hospital and Institute, Beijing 100142, China

## Abstract

**Purpose:**

This study aimed to assess the efficacy of dual-tracer [^68^Ga-DOTA-somatostatin receptor analogs (SSAs) and ^18^F-fluorodeoxyglucose (FDG)] positron emission tomography/computed tomography (PET/CT) imaging for detecting bone metastases (BMs) in patients with gastroenteropancreatic neuroendocrine neoplasms (GEP-NENs).

**Methods:**

We retrospectively enrolled 74 GEP-NEN patients with BMs from two centers, who underwent dual-tracer PET/CT from January 2014 to March 2021. We compared and analyzed effectiveness of the dual PET/CT imaging techniques on the BMs, based on ^18^F-FDG and ^68^Ga-DOTA-SSAs. Specifically, we analyzed the imaging results using *χ*^2^ tests for classification variables, paired-sample tests for number of BMs, Wilcoxon's signed rank test for number of lesions, and the Kruskal–Wallis test for standard uptake value (SUV) ratio comparison. The correlation of dual-tracer SUVmax with Ki-67 index was analyzed by Spearman's correlation coefficient.

**Results:**

The detection efficiencies of dual-tracer PET/CT imaging in patients with different pathologies showed discordant for detecting liver metastases and BMs in group neuroendocrine tumor (NET) G3, ^68^Ga-DOTA-SSAs was better at detecting BMs for NET G3 (*P*=0.049 for SUV_T/B_ and *P*=0.026 for the number of metastatic lesions). In addition, statistical significance was found among osteogenesis group, osteolysis group, and the no-change group (for bone SUV_T/B_ value detected by ^18^F-FDG and Ki-67 index, osteogenesis group < osteolysis group; for bone SUV_T/B_ detected by ^68^Ga-DOTA-SSAs, osteogenesis group > the no-change group). What is more, liver and bone SUVmax and Ki-67 index were positively correlated in ^18^F-FDG imaging (*P* < 0.001 for liver; *P*=0.002 for bone), and negatively correlated in ^68^Ga-DOTA-SSAs imaging (*P* < 0.001 for liver; *P*=0.039 for bone).

**Conclusions:**

^68^Ga-DOTA-SSAs was superior to ^18^F-FDG for detecting BMs in NET G1/G2 (well and moderately differentiated NETs), as well as in NET G3 (poorly differentiated NETs). Relatively good differentiation was observed in the osteogenesis group. In addition, dual-tracer PET/CT imaging results were observably correlated with tumor differentiation.

## 1. Introduction

Gastroenteropancreatic neuroendocrine neoplasms (GEP-NENs) are heterogeneous neoplasms that show neuroendocrine differentiation, with peculiar histomorphological and clinical features [1]. NENs are usually considered rare cancers (∼0.5% of all malignancies); however, the apparent incidence of NENs has increased rapidly and gained recent attention in line with the development of modern imaging techniques [2, 3]. Distant metastases are often observed at diagnosis in patients with GEP-NENs, most frequently in the liver [3]. Bone metastases (BMs), frequently accompanied by the development of liver metastases (LMs), are usually considered to be a late event in NENs and predictive of a poor prognosis; however, tumor grading and evaluation of the biological characteristics, they often remain undetected [4–6]. This may be due to the limitations of previous imaging methods and the longer survival of NEN patients. BMs may present with pain as a main symptom, while other common skeletal-related events include pathological bone fractures, spinal cord compression, and hypercalcemia, which can have a strong impact on the patient's quality of life [4]. The patient's general deterioration may also lead to treatment discontinuation, resulting in tumor progression, in patients with GEP-NENs. In addition, BMs are a significant prognostic factor affecting overall survival, which is significantly reduced in patients with BMs compared with those with other distant metastases [7]. It is therefore necessary to detect and evaluate bone involvement as early as possible.

In the past, the diagnosis of NENs was relied on structural imaging, including computed tomography (CT) and magnetic resonance imaging (MRI), which was less effective. The combined use of single-photon emission computed tomography (SPECT) and CT strongly supports the molecular imaging of NENs with somatostatin receptor radiopharmaceuticals; the fusion images provide higher specificity and accurate localization of neuroendocrine tumors (NETs) [8]. Positron emission tomography (PET), the more advanced application of nuclear medicine imaging, has more extensive use over SPECT in the diagnostics for NETs, e.g., PET has higher spatial resolution and unique sensitivity to visualize in vivo cellular metabolism, in addition, PET has advantages on the inherently quantitative nature [9]. PET/CT-based molecular imaging has become indispensable for the management of GEP-NENs, and NEN receptor expression or metabolism can be characterized by employing different PET radiopharmaceuticals. Currently used radiopharmaceuticals include ^18^F-fluorodeoxyglucose (FDG) and ^68^Ga somatostatin receptor analogs (SSAs), including ^68^Ga-DOTA-Tyr3-octreotate (^68^Ga-DOTA-TATE), ^68^Ga-DOTA-D-Phe1-Tyr3-octreotide (^68^Ga-DOTA-TOC), and ^68^Ga-DOTA-1-Nal3-octreotide (^68^Ga-DOTA-NOC), which are targeted to somatostatin receptors [10–12]. ^68^Ga-DOTA-TATE and ^68^Ga-DOTA-TOC showed high affinity for SSTR2 and SSTR5, which are main SSTR subtypes found in NENs. ^68^Ga-DOTA-NOC targeted a wider range of somatostatin subtype receptors, including SSTR2, SSTR3, and SSTR5. Despite differences in receptor affinity, there is no clear evidence showing any of these imaging agents a convincing advantage. These ^68^Ga-DOTA-SSAs have frequently been used for staging, restaging, and therapy response assessment, as well as for selecting patients eligible for radioligand therapy [13–15].

The two types of tracers show complementary characteristics and have thus been compared and investigated in previous studies [16–21]. However, few studies [16] have focused on the detection or evaluation of GEP-NENs with BMs using dual-tracer PET/CT imaging, and the sample sizes were too small to explore the correlation between imaging and pathological tumor changes. The current two-center retrospective head-to-head study aimed to evaluate the detection efficiency of dual-tracer PET/CT imaging and the correlation between imaging results and tumor proliferation in patients with histologically proven GEP-NENs with BMs.

## 2. Materials and Methods

### 2.1. Patient Population

We collected data from GEP-NEN patients with BMs who underwent dual-tracer PET/CT (^68^Ga-DOTA-SSAs and ^18^F-FDG) over the same period from January 2014 to March 2021. We have 74 patients of GEP-NENs with BMs included in our retrospective analysis. The overall median age of patients was 55.93 (±11.025, range 26–77), and the number of male patients is 47 (63.51%). According to the recent consensus statements from the European Neuroendocrine Tumor Society, all the specimens were pathologically confirmed and graded based on the mitotic count and Ki-67 index. Molecular differences, including immunohistochemical staining of TP53, RB1, ATRX, and DAXX, were also considered when identifying NET G3 and neuroendocrine carcinoma (NEC) tumors [22].

Patient data were obtained from the Department of Nuclear Medicine, Peking University Cancer Hospital and the Institute and Department of Nuclear Medicine, Nanjing First Hospital. All BMs were confirmed by pathology or clinical follow-up. Dual-tracer PET/CT examinations were performed within a maximum interval of 4 weeks (median 7.75 days), which was considered sufficiently short given the relatively slow progression of NENs. No patients were treated during this interval.

This study was approved by the Ethics Committee of Peking University Cancer Hospital and Nanjing First Hospital. All subjects signed informed consent forms before participating in this study.

### 2.2. Image Acquisition

PET/CT scans were performed using a Siemens PET/CT scanner (Biograph64; Siemens, Erlangen, Germany) at the Nuclear Medicine Department of Peking University Cancer Hospital, or a uMI 780 PET/CT scanner (United Imaging Healthcare, Shanghai, China) at the Nuclear Medicine Department of Nanjing First Hospital.

Patients fasted for at least 6 hr before PET/CT scanning. Images were acquired 60 ± 10 min after the injection of ^18^F-FDG (3.7 MBq/kg) or ^68^Ga-DOTA-SSAs (100–200 MBq). Blood glucose levels were checked before ^18^F-FDG injection and fasting blood glucose levels were <11 mmol/L in all patients.

The PET and CT acquisition range was consistent, and whole-body scanning (skull top to mid-thigh) was performed in the supine position with the following parameters: CT exposure factors 120 kV and 100 mA, scanning layer thickness 3 mm, pitch 0.8 mm, and nine beds collected by PET (Siemens PET/CT), or CT exposure factors 120 kV and 100–500 mA, scanning layer thickness 5 mm, pitch 0.9875 mm, and four beds collected by PET (uMI 780 PET/CT). The ordered subsets expectation maximization method was used for PET image reconstruction. The numbers of iterations and subsets of iterations were 3 and 33, respectively, for the Siemens Inveon PET/CT, and 2 and 20 for the uMI 780 PET/CT. CT images were used to correct the PET emission data for photon attenuation.

### 2.3. Image Analysis

Two senior nuclear medicine physicians read the imaging data for all patients separately. Manually defined circular regions of interest were drawn to measure the maximum standard uptake value (SUVmax) for each lesion. The diagnostic results of dual-tracer PET/CT were scored as positive if the highest radiation uptake in all lesions was higher than the normal liver background. BMs were defined as abnormal bone density (except for benign bone diseases such as degenerative degeneration) with higher local radioactivity distribution than the surrounding normal bone background. SUV_T/B_ denotes the target-to-background SUV ratio. SUVmax values were measured with a diameter of 2 cm. The SUVmax of normal bone was measured in the second lumbar vertebral body, or in other thoracic or lumbar vertebrae if the second lumbar spine had BMs, and normal bone in the axial skeleton was measured in the case of diffuse multiple bone lesions. The SUVmax of normal liver was measured in the right liver lobe in a relatively large plane while avoiding large blood vessels in the liver parenchyma, and in other normal liver parenchyma in patients with multiple metastases in the right lobe. 

### 2.4. Statistical Analysis

Normally distributed variables such as age were expressed as mean ± standard deviation or range. Other patient characteristics were recorded as absolute numbers or percentages. Differences between dual-tracer imaging groups in terms of classification variables were analyzed by *χ*^2^ tests and numbers of BMs in each site were compared by paired samples tests. SUV_T/B_ and the number of lesions were compared using Wilcoxon's signed rank test, the difference in SUV_T/B_ between groups was assessed by the Kruskal–Wallis test, and the correlation between dual-tracer SUVmax values and Ki-67 index was calculated using Spearman's correlation coefficient. A *P* value < 0.05 in two-tailed tests was considered statistically significant. Statistical analysis was performed using SPSS version 24.0 software (IBM Corp., Armonk, NY).

## 3. Results

### 3.1. Patient Characteristics

A total of 74 patients with pathologically confirmed GEP-NENs with BMs were included in this retrospective analysis. Among all the cases, 5 were confirmed pathologically and 69 were further confirmed by bone lesion progression or other imaging during follow-up. The basic characteristics of the patients are summarized in Table 1. Altogether, 29, 17, and 28 patients underwent surgical resection, endoscopic procedure, and puncture biopsy, respectively. Pathological evaluation showed that 3 patients (4.05%) had G1, 47 (63.51%) had G2, and 12 (16.22%) had NET G3, and 12 patients (16.22%) had NEC. For statistical analysis, we integrated G1/G2 into one group and included NET G3 and NEC as two additional groups.

The interval time between pathological examination and imaging was 509.23 days (range, 1–2,570 days). The primary tumor locations were the stomach, intestine, pancreas, esophagus, biliary tract, and unknown (Table 1). 32 patients (43.24%) underwent resection of the primary lesion and 10 (13.51%) underwent partial hepatectomy of LMs before PET/CT examination. 31, 6, 8, 25, and 21 patients received chemotherapy, radiotherapy, interventional therapy, octreotide therapy, and peptide receptor radionuclide therapy, respectively. In total, 69 patients had LMs, 50 had lymph node involvement, and 9 patients had other distant metastases, including lung, kidney, paranephros, pelvic metastases. In total, 15 patients (20.27%) had a medical history of bone pain, of whom 10 (13.51%) had required additional analgesics for pain relief. Considering the CT findings, 41 patients mainly had osteogenesis, 18 mainly had osteolysis, and 15 patients mainly had no changes.

### 3.2. Detection Efficiencies of Dual-Tracer PET/CT Imaging

It turned out that the dual-tracer imaging did not show consistent results. ^68^Ga-DOTA-SSAs imaging was positive in 61 cases and negative in 13 cases, while ^18^F-FDG imaging was positive in 42 cases and negative in 32 cases (*χ*^2^ = 8.121, *P*=0.004).

### 3.3. Detection Numbers

The distribution and number of BMs detected by dual-tracer imaging are demonstrated in Figure 1. ^68^Ga-DOTA-SSAs detected more patients with BMs for all sites, including spine, pelvis, ribs, sternum-clavicle-scapula, proximal limbs, and skull, compared with ^18^F-FDG (*t* = 6.435, *P*=0.001).

### 3.4. SUV Value Comparison

We compared the detection efficiencies of dual-tracer PET/CT imaging in patients with different pathologies (Table 2). Patients were divided into three groups: G1 + G2 (well and moderately differentiated NETs), NET G3 (poorly differentiated NETs), and NEC. SUV_T/B_ and the number of metastatic lesions detected by each tracer PET/CT were observed for LMs and BMs.

^68^Ga-DOTA-SSAs imaging performed better in patients with lower tumor proliferation while ^18^F-FDG imaging was better in patients with higher proliferation. ^68^Ga-DOTA-SSAs imaging achieved better detection results in group G1 + G2 in terms of numbers of lesions and LMs and BMs SUV_T/B_ ratios than ^18^F-FDG imaging (*P* < 0.05 for all items).

However, the efficiency of dual-tracer imaging for detecting LMs and BMs in group NET G3 was discordant: ^18^F-FDG PET/CT showed slightly superior detection efficiency for LMs while ^68^Ga-DOTA-SSAs imaging showed significantly better detection of BMs (shown in the penult row of Table 2). The imaging advantages of ^68^Ga-DOTA-SSAs for BM lesions in patients with NET G3 are illustrated in a patient with liver, lymph node, and BMs of an unknown primary in Figure 2.

^68^Ga-DOTA-SSAs imaging also showed better results for BM detection in patients with NEC, but the difference was not significant, while ^18^F-FDG PET/CT was significantly better than ^68^Ga-DOTA-SSAs imaging for detecting LMs.

### 3.5. Correlation between Dual-Tracer PET/CT Imaging and Tumor Differentiation

#### 3.5.1. Correlation between CT Appearance and Tumor Differentiation

The patients were divided into three groups according to the changes in bone density on CT. There were 41 cases in the osteogenesis group, 18 in the osteolysis group, and 15 in the no-change group.

As shown in Figure 3, patients in the osteogenesis group had higher BM SUV_T/B_ values than those in the no-change group for ^68^Ga-DOTA-SSAs imaging (Figure 3(a), *P*=0.046). However, for ^18^F-FDG PET/CT the value was lower in the osteogenesis group compared with the osteolysis group (Figure 3(b), *P*=0.021). In addition, we explored tumor differentiation as determined by Ki-67 index (Figure 3(c)), which showed that patients in the osteogenesis group had relatively higher tumor differentiation (*P*=0.048). A patient with a rectal G2 and osteogenesis, with a higher SUV_T/B_ on ^68^Ga-DOTA-SSAs PET/CT and lower bone SUV_T/B_ on ^18^F-FDG PET/CT, is shown in Figure 4.

#### 3.5.2. Correlation between SUV Value and Tumor Differentiation for Each Imaging Method

The SUV value differed significantly across histologic subtypes (Figure 5). In pairwise comparisons, the LMs SUV_T/B_ and BMs SUV_T/B_ for ^18^F-FDG were significantly lower in the G1 + G2 group compared with the NET G3 group (*P* < 0.005 for both comparisons), and the LMs SUV_T/B_ for ^68^Ga-DOTA-SSAs was significantly higher in the G1 + G2 compared with the NET G3 group (*P* < 0.005). The BMs SUV_T/B_ of ^68^Ga-DOTA-SSAs had an advantage in group G1 + G2 compared with group NET G3, but the difference was not significant (*P*=0.066). The LMs SUV_T/B_ and BMs SUV_T/B_ were significantly lower in the G1 + G2 group compared with the NEC group for ^18^F-FDG but significantly higher for ^68^Ga-DOTA-SSAs imaging (*P* < 0.005 for both comparisons). There was no difference between the NET G3 and NEC groups in terms of SUV_T/B_ for either tracer.

### 3.6. Correlation between SUVmax and Ki67 Index for Each Imaging Method

The SUVmax for dual-tracer PET/CT imaging was significantly correlated with tumor differentiation. There were significant positive correlations between the SUVmax values of both LMs and BMs detected by ^18^F-FDG and Ki-67 index (Spearman's *r* = 0.452, *P* < 0.001; Spearman's *r* = 0.355, *P*=0.002, respectively), but significant negative correlations in ^68^Ga-DOTA-SSAs imaging (Spearman's *r *= −0.440, *P* < 0.001; Spearman's *r *= −0.240, *P*=0.039, respectively) (Figure 6).

## 4. Discussion

This study aimed to evaluate the efficacy of dual-tracer PET/CT imaging for detecting BMs in patients with GEP-NENs and to investigate the correlation between the SUV value and tumor differentiation for each tracer. ^68^Ga-DOTA-SSA imaging was superior to ^18^F-FDG in terms of the number of detected lesions and radioactivity uptake by lesions in patients with well-differentiated GEP-NENs. In addition, ^68^Ga-DOTA-SSAs detected a higher bone SUV_T/B_ in the osteogenesis group. Furthermore, the detection efficiency of ^68^Ga-DOTA-SSAs differed between LMs and BMs in the NET G3 group, with LMs detected slightly better by ^18^F-FDG PET/CT and BMs detected better by ^68^Ga-DOTA-SSAs. The number of detected BMs and the bone SUV_T/B_ were significantly higher according to ^68^Ga-DOTA-SSAs, further explaining the advantage of ^68^Ga-DOTA-SSAs imaging for the detection of BMs in patients with GEP-NENs.

We considered the possible reasons for the advantages of ^68^Ga-DOTA-SSAs imaging for detecting BMs in patients with GEP-NENs. First, ^68^Ga-DOTA-SSAs imaging detects radioactivity uptake by the tumor lesions, due to the relatively low-level blood pool and the background SUV of normal bone, making it easy to detect small lesions. Second, ^68^Ga-DOTA-SSAs is a functional imaging agent that binds somatostatin receptors expressed on NET cells with variable affinity, making it useful for not only detecting NET lesions but also providing valuable diagnostic information on the expression of tumor cell receptors [23]. This might explain the higher uptake by potential BMs. Finally, apart from malignant lesions, ^18^F-FDG PET/CT has also been found to detect benign skeletal lesions [24, 25]. Considering the glucose metabolism-imaging mechanism of ^18^F-FDG, its high sensitivity and low specificity may account for false positive diagnoses in cases of trauma, infection, inflammation, and other benign conditions. In contrast, ^68^Ga-DOTA-SSAs imaging is less-affected than ^18^F-FDG PET/CT by such conditions, leading to better specificity and detection accuracy of ^68^Ga-DOTA-SSAs for BMs [26]. Notably, a previous study came to a similar conclusion regarding the advantages of ^68^Ga-DOTA-SSAs for detecting BMs but failed to demonstrate a statistical difference [17].

CT performance of BMs also correlated with pathological tumor changes. The mechanism responsible for BMs is currently unclear, but recent studies [27] suggested the existence of related regulatory effects between tumor cells and changes in the bone microenvironment, even in the absence of clinical symptoms of BMs. For example, the ratio of RANK-ligand/osteoprotegerin produced by osteoblasts is unbalanced, leading to changes in bone remodeling [28]. Damage to this pathway is common to different types of tumors, including GEP-NENs and bronchopulmonary NENs [29]. In the current retrospective study, we analyzed BMs of GEP-NENs from a clinical perspective, to clarify the association between GEP-NEN tumor differentiation and CT imaging findings. We observed that the Ki-67 index was significantly lower in patients with osteogenesis, while there were no significant differences in patients in the osteolysis and no-change groups. The use of appropriate imaging technology may allow the earlier diagnosis of BM, thus preventing the development of skeletal-related events and guaranteeing patient quality of life. We suggest that the CT findings of osteogenic changes in BMs may indicate that the GEP-NENs are well differentiated, thus providing promising evidence for the differentiation of GEP-NENs.

In this study, we observed a significant correlation between dual-tracer PET/CT imaging and tumor differentiation. ^18^F-FDG performs well for the evaluation and management of high-grade NENs (poorly differentiated and aggressive) [30], but has limitations for the determination of metastatic lesions in well-differentiated NENs, because ^18^F-FDG PET/CT is positively correlated with the degree of tumor malignancy and is less sensitive in well-differentiated NETs. There is thus a significant positive correlation between the SUVmax of BMs detected by ^18^F-FDG and Ki-67 index [31]. In contrast, ^68^Ga-DOTA-SSAs imaging is better at detecting low-grade NENs, with a negative correlation that presents complementary characteristics for the diagnosis and staging of NENs and the selection of an appropriate treatment regimen [32]. “Flip-flop” was a phenomenon proposed in thyroid carcinoma to describe an inverse relationship between iodine and ^18^F-FDG accumulation: thyroid cancer cells tend to lose radioiodine avidity, and start to take up ^18^F-FDG when tumor get differentiated [33]. This phenomenon has also been adopted prevalently in NEN: a poorer tumor differentiation exhibits a decreased DOTATATE expression and an increased FDG uptake [34]. However, it should be noted that this dedifferentiation process represents a spectrum rather than a yes/no question; quite a few patients demonstrated features of both SSTR high expression and FDG high uptake [35]. Thus, the integration of these two tracers may provide a more comprehensive imaging strategy [36].

The current study conducted more investigations than previous studies of BMs in patients with GEP-NENs. For example, Scharf et al. [7] examined the incidence and clinical and prognostic impacts of BMs in patients with NENs but failed to provide any imaging-related analysis of the cohort. Another recent study [37] confirmed the high sensitivity of ^68^Ga-DOTATOC-PET/CT for detecting vertebral metastases in a larger cohort of NEN patients (*n* = 535), but the authors failed to compare the morphological and functional imaging results. Zhang et al. [16] demonstrated the advantages of ^68^Ga-DOTATATE in dual-tracer imaging (better performance in 62.5% of cases) in patients with GEP-NENs, but the sample size was very small (*n* = 8) and there was analysis of the efficacy of dual-tracer imaging for detecting BMs in relation to tumor differentiation. To the best of our knowledge, the current study provides the first evidence for the performance of dual-tracer imaging with ^68^Ga-DOTA-SSAs and ^18^F-FDG in patients with well, moderately, and poorly differentiated NENs accompanied by BMs. In addition, we analyzed cases from two centers over 7 years, leading to more representative conclusions. In recent years, sodium fluoride labeled ^18^F (NaF) PET/CT tends to be a useful alternative to detect primary malignant bone tumors and BMs [38]. Since there are few related studies for patients with GEP-NENs using NaF, in the future work we will pay more attention to this research direction. Another promising new tracer of NENs for PET/CT imaging is ^68^Ga-DOTA-JR11, which performs better in detecting LMs while worse in BMs compared with ^68^Ga-DOTATATE [39]. An emerging and promising radiotracer for PET/CT imaging is [^68^Ga]Ga-FAPI, which indicated high uptake of [^68^Ga]Ga-FAPI in NET of different origins in several case reports [40, 41]. Although these studies are very preliminary, they may facilitate novel diagnostic as well as therapeutic options for NEN patients, and further studies are needed to better ascertain their clinical value.

The current study also had some limitations. The sample size was small for the NET G3 and NEC groups. Besides, despite using SUV_T/B_ to reduce the impacts caused by different tomographs from two centers, we should not ignore this data distribution problem in the analysis. In addition, this retrospective analysis has an inherent limitation: conclusions need to be confirmed in future randomized controlled studies.

## 5. Conclusion

In this study, we compared the multidimensional performances of dual-tracer PET/CT imaging in GEP-NEN patients with BMs. ^68^Ga-DOTA-SSAs was superior to ^18^F-FDG for detecting BMs in terms of the number and SUV_T/B_ of the detected lesions. We analyzed patients with tumors with different degrees of differentiation separately, including G1, G2, and G3 NET groups. We also observed that patients with osteogenesis showed relatively well-differentiated lesions, which might provide promising evidence for NEN differentiation. In addition, dual-tracer PET/CT imaging showed strong complementary correlations with tumor differentiation. Further randomized controlled trials are needed to explore the detection advantages of dual-tracer imaging in patients GEP-NENs with BMs.

## Figures and Tables

**Figure 1:** Distributions of bone metastases in the spine, pelvis, ribs, sternum-clavicle-scapula, proximal limbs, and skull detected in dual-tracer imaging (*χ*^2^ tests for comparison between ^68^Ga-DOTA-SSAs and ^18^F-FDG groups, *P* < 0.01 for each group).

**Figure 2:** Dual-tracer imaging in a 46-year-old woman with NET G3 (Ki-67 index 22%) accompanied by liver, lymph node, and bone metastases of unknown primary origin: (a1, a2) Maximum intensity projection of dual-tracer imaging; (b1, b2) Sternum lesion with somatostatin receptor (SSTR) expression on ^68^Ga-DOTA-SSAs PET/CT but no bone metastases were detected by ^18^F-FDG PET/CT; (c1, c2) ^18^F-FDG PET/CT imaging of liver lesions showing liver metastases (LMs) with higher FDG metabolism, while ^68^Ga-DOTA-SSAs PET/CT imaging showed LMs with lower SSTR expression.

**Figure 3:** Correlation between computed tomography appearance and tumor differentiation: (a) bone metastases (BMs) SUVT/B detected by ^68^Ga-DOTA-SSAs; (b) BMs SUVT/B detected by ^18^F-FDG; (c) Ki-67 index. Patients were divided into osteogenesis, osteolysis, and no-change groups. ^*∗*^Kruskal–Wallis test for comparison between osteogenesis and osteolysis groups; ^#^Kruskal–Wallis test for comparison between osteogenesis and no change groups.

**Figure 4:** Dual-tracer imaging in a 57-year-old man with rectal NET G2 (Ki-67 index 3%), accompanied by liver, lymph node, and bone metastases. The patient suffered from systemic diffuse bone metastases, including in the spine, pelvis, ribs, sternum-clavicle-scapula, proximal limbs, and skull. Computed tomography findings mainly manifested osteogenesis changes. b1 and c1 show more bone lesions than ^18^F-FDG PET/CT imaging. (a–c) Maximum intensity projection, osteogenesis in the pelvis, and osteogenesis in the spine, respectively, detected by dual-tracer imaging.

**Figure 5:** Detection efficiency of dual-tracer PET/CT imaging in different pathological groups. ^*∗*^Kruskal–Wallis test for comparison between G1 + G2 and G3 groups; ^#^Kruskal–Wallis test for comparison between G1 + G2 and NEC groups.

**Figure 6:** Correlation between maximum standard uptake value and Ki-67 index in liver and bone in single-tracer imaging.

**Table 1:** Patient characteristics (*n* = 74).

Basics	Total	G1 + G2	NET G3	NEC	*P*
*N* (%)	74	50	12	12	
Age at image (mean ± SD)	55.93 ± 11.025	55.66 ± 10.817	51.58 ± 8.028	61.42 ± 12.930	0.086
Sex, M/F (%)	47/27 (63.51/36.49)	32/18 (64.00/36.00)	8/4 (66.67/33.33)	7/5 (58.33/41.67)	0.905

Primary sites (*n*, %)					
Stomach	6 (8.11)	3 (6)	1 (8.33)	2 (16.67)	0.546
Intestine	34 (45.95)	28 (56)_a_	4 (33.33)_b_	2 (16.67)_c_	0.028
Pancreas	26 (35.14)	17 (34)	4 (33.33)	5 (41.67)	0.933
Esophagus	3 (4.05)	1 (2)		2 (16.67)	0.133
Biliary tract	2 (2.70)		1 (8.33)	1 (8.33)	0.102
Unknown primary origin	3 (4.05)	1 (2)	2 (16.67)		0.133

Other extra-osseous metastases (*n*, %)					
Liver metastases	69 (93.24)	48 (96)	11 (91.67)	10 (83.33)	0.482
Lymph node metastases	50 (67.57)	36 (72)	5 (41.67)	9 (75)	0.134

Symptoms	15 (20.27)	7 (14)	3 (25)	5 (41.67)	0.073

CT findings (*n*, %)					
Osteogenesis	41 (55.41)	34 (68)_a_	5 (41.67)_b_	2 (16.67)_c_	0.003
Osteolysis	18 (24.32)	9 (18)	5 (4.05)	4 (33.33)	0.245
No change	15 (20.27)	7 (14)_b_	2 (16.67)_b_	6 (50)_a_	0.026

CT, computed tomography; M/F, male/female; _a,__b,_ and _c_ (where _a_>_b_>_c_) mark statistically significant differences between each group.

**Table 2:** Comparison of the detection SUV value of ^18^F-FDG PET/CT and ^68^Ga-DOTA-SSAs PET/CT imaging.

Part	Liver metastases					Bone metastases				
	*N*	Type	^18^F-FDG	^68^Ga-DOTA-SSAs	Wilcoxon *P*	*N*	Type	^18^F-FDG	^68^Ga-DOTA-SSAs	Wilcoxon *P*
Total	69	SUV_T/B_	2.29 ± 1.48	4.92 ± 4.50	≤0.001	74	SUV_T/B_	3.03 ± 2.64	25.70 ± 24.26	≤0.001
		Amount	10.67 ± 23.05	21.53 ± 31.41	0.010		Amount	9.81 ± 22.89	25.91 ± 36.87	≤0.001
G1 + G2	48	SUV_T/B_	1.70 ± 0.78	6.11 ± 4.83	≤0.001	50	SUV_T/B_	2.04 ± 1.33	30.29 ± 25.90	≤0.001
		Amount	5.44 ± 14.50	22.77 ± 30.53	≤0.001		Amount	7.36 ± 20.24	25.62 ± 36.39	≤0.001
G3	11	SUV_T/B_	3.45 ± 2.17	2.31 ± 2.34	0.110	12	SUV_T/B_	4.32 ± 2.95	16.88 ± 15.75	0.049
		Amount	17.00 ± 28.79	16.64 ± 29.22	0.722		Amount	13.75 ± 28.50	24.50 ± 37.10	0.026
NEC	10	SUV_T/B_	3.98 ± 1.21	2.26 ± 1.77	0.280	12	SUV_T/B_	5.50 ± 3.95	12.76 ± 16.39	0.272
		Amount	29.90 ± 37.90	22.70 ± 40.92	0.025		Amount	15.00 ± 28.23	22.33 ± 36.81	0.531

## Data Availability

The datasets used and/or analyzed during the current study are available from the corresponding author on reasonable request.

## Abbreviations

BMs: Bone metastases
FDG: ^18^F-fluorodeoxyglucose
^68^Ga-DOTA-NOC: ^68^Ga-DOTA-1-Nal3-octreotide
^68^Ga-DOTA-TATE: ^68^Ga-DOTA-Tyr3-octreotate
^68^Ga-DOTA-TOC: ^68^Ga-DOTA-D-Phe1-Tyr3-octreotide
GEP-NENs: Gastroenteropancreatic neuroendocrine neoplasms
LMs: Liver metastases
PET/CT: Positron emission tomography/computed tomography.

## References

[1] Faggiano A., Ferolla P., Grimaldi F. (2012). Natural history of gastro-entero-pancreatic and thoracic neuroendocrine tumors. Data from a large prospective and retrospective Italian epidemiological study: the NET management study. *Journal of Endocrinological Investigation*.

[2] Yao J. C., Hassan M., Phan A. (2008). One hundred years after “Carcinoid”: epidemiology of and prognostic factors for neuroendocrine tumors in 35,825 cases in the United States. *Journal of Clinical Oncology*.

[3] Hallet J., Law C. H. L., Cukier M., Saskin R., Liu N., Singh S. (2015). Exploring the rising incidence of neuroendocrine tumors: a population-based analysis of epidemiology, metastatic presentation, and outcomes. *Cancer*.

[4] Kos-Kudła B., O’Toole D., Falconi M. (2010). ENETS consensus guidelines for the management of bone and lung metastases from neuroendocrine tumors. *Neuroendocrinology*.

[5] Coleman R. E. (2001). Metastatic bone disease: clinical features, pathophysiology and treatment strategies. *Cancer Treatment Reviews*.

[6] Van Loon K., Zhang L., Keiser J. (2015). Bone metastases and skeletal-related events from neuroendocrine tumors. *Endocrine Connections*.

[7] Scharf M., Petry V., Daniel H., Rinke A., Gress T. M. (2018). Bone metastases in patients with neuroendocrine neoplasm: frequency and clinical, therapeutic, and prognostic relevance. *Neuroendocrinology*.

[8] Fuccio C., Spinapolice E. G., Chondrogiannis S. (2013). Evolving role of SPECT/CT in neuroendocrine tumors management: staging, treatment response, and follow-up. *Clinical Nuclear Medicine*.

[9] Pfeifer A., Knigge U., Binderup T. (2015). ^64^Cu-DOTATATE PET for neuroendocrine tumors: a prospective head-to-head comparison with ^111^In-DTPA-octreotide in 112 patients. *Journal of Nuclear Medicine*.

[10] Deppen S. A., Liu E., Blume J. D. (2016). Safety and efficacy of ^68^Ga-DOTATATE PET/CT for diagnosis, staging, and treatment management of neuroendocrine tumors. *Journal of Nuclear Medicine*.

[11] Buchmann I., Henze M., Engelbrecht S. (2007). Comparison of ^68^Ga-DOTATOC PET and ^111^In-DTPAOC (Octreoscan) SPECT in patients with neuroendocrine tumours. *European Journal of Nuclear Medicine and Molecular Imaging*.

[12] Krausz Y., Freedman N., Rubinstein R. (2011). ^68^Ga-DOTA-NOC PET/CT imaging of neuroendocrine tumors: comparison with ^111^In-DTPA-octreotide (OctreoScan®). *Molecular Imaging and Biology*.

[13] Muffatti F., Partelli S., Cirocchi R. (2019). Combined ^68^Ga-DOTA-peptides and ^18^F-FDG PET in the diagnostic work-up of neuroendocrine neoplasms (NEN). *Clinical and Translational Imaging*.

[14] Urso L., Nieri A., Rambaldi I. (2022). Radioligand therapy (RLT) as neoadjuvant treatment for inoperable pancreatic neuroendocrine tumors: a literature review. *Endocrine*.

[15] Binderup T., Knigge U., Loft A., Federspiel B., Kjaer A. (2010). ^18^F-fluorodeoxyglucose positron emission tomography predicts survival of patients with neuroendocrine tumors. *Clinical Cancer Research*.

[16] Zhang P., Yu J., Li J. (2018). Clinical and prognostic value of PET/CT imaging with combination of ^68^Ga-DOTATATE and ^18^F-FDG in gastroenteropancreatic neuroendocrine neoplasms. *Contrast Media & Molecular Imaging*.

[17] Nilica B., Waitz D., Stevanovic V. (2016). Direct comparison of ^68^Ga-DOTA-TOC and ^18^F-FDG PET/CT in the follow-up of patients with neuroendocrine tumour treated with the first full peptide receptor radionuclide therapy cycle. *European Journal of Nuclear Medicine and Molecular Imaging*.

[18] Paiella S., Landoni L., Tebaldi S. (2022). Dual-tracer (^68^Ga-DOTATOC and ^18^F-FDG-)-PET/CT scan and G1-G2 nonfunctioning pancreatic neuroendocrine tumors: a single-center retrospective evaluation of 124 nonmetastatic resected cases. *Neuroendocrinology*.

[19] Panagiotidis E., Alshammari A., Michopoulou S. (2017). Comparison of the impact of ^68^Ga-DOTATATE and ^18^F-FDG PET/CT on clinical management in patients with neuroendocrine tumors. *Journal of Nuclear Medicine*.

[20] Urso L., Panareo S., Castello A. (2022). Glucose metabolism modification induced by radioligand therapy with [^177^Lu]Lu/[^90^Y]Y-DOTATOC in advanced neuroendocrine neoplasms: a prospective pilot study within FENET-2016 trial. *Pharmaceutics*.

[21] Oh S., Prasad V., Lee D. S., Baum R. P. (2011). Effect of peptide receptor radionuclide therapy on somatostatin receptor status and glucose metabolism in neuroendocrine tumors: intraindividual comparison of Ga-68 DOTANOC PET/CT and F-18 FDG PET/CT. *International Journal of Molecular Imaging*.

[22] Shah M. H., Goldner W. S., Benson A. B. (2021). Neuroendocrine and adrenal tumors, version 2.2021, NCCN clinical practice guidelines in oncology. *Journal of the National Comprehensive Cancer Network*.

[23] von Falck C., Boerner A. R., Galanski M., Knapp W. H. (2007). Neuroendocrine tumour of the mediastinum: fusion of ^18^F-FDG and ^68^Ga-DOTATOC PET/CT datasets demonstrates different degrees of differentiation. *European Journal of Nuclear Medicine and Molecular Imaging*.

[24] Feldman F., van Heertum R., Manos C. (2003). ^18^FDG PET scanning of benign and malignant musculoskeletal lesions. *Skeletal Radiology*.

[25] Kwee T. C., de Klerk J. M. H., Nix M., Heggelman B. G. F., Dubois S. V., Adams H. J. A. (2017). Benign bone conditions that may be FDG-avid and mimic malignancy. *Seminars in Nuclear Medicine*.

[26] Naswa N., Sharma P., Gupta S. K. (2014). Dual tracer functional imaging of gastroenteropancreatic neuroendocrine tumors using ^68^Ga-DOTA-NOC PET-CT and ^18^F-FDG PET-CT: competitive or complimentary?. *Clinical Nuclear Medicine*.

[27] Kaplan R. N., Rafii S., Lyden D. (2006). Preparing the “soil”: the premetastatic niche. *Cancer Research*.

[28] Tat S. K., Padrines M., Theoleyre S. (2006). OPG/membranous—RANKL complex is internalized via the clathrin pathway before a lysosomal and a proteasomal degradation. *Bone*.

[29] Milone F., Pivonello C., Cariati F. (2013). Assessment and clinical implications of RANK/RANKL/OPG pathway as markers of bone tumor progression in patients with NET harboring bone metastases. *Biomarkers*.

[30] Howe J. R. (2015). The supporting role of ^18^FDG-PET in patients with neuroendocrine tumors. *Annals of Surgical Oncology*.

[31] Yu J., Li N., Li J. (2019). The correlation between [^68^Ga]DOTATATE PET/CT and cell proliferation in patients with GEP-NENs. *Molecular Imaging and Biology*.

[32] Bauckneht M., Albano D., Annunziata S. (2020). Somatostatin receptor PET/CT imaging for the detection and staging of pancreatic NET: a systematic review and meta-analysis. *Diagnostics*.

[33] Feine U., Lietzenmayer R., Hanke J. P., Wöhrle H., Müller-Schauenburg W. (1995). ^18^FDG whole-body PET in differentiated thyroid carcinoma. Flipflop in uptake patterns of ^18^FDG and ^131^I. *Nuklearmedizin*.

[34] Hofman M., Pacak K., Taïeb D. (2017). Principles and application of molecular imaging for personalized medicine and guiding interventions in neuroendocrine tumors. *Diagnostic and Therapeutic Nuclear Medicine for Neuroendocrine Tumors. Contemporary Endocrinology*.

[35] Pattison D. A., Hofman M. S. (2015). Role of fluorodeoxyglucose PET/computed tomography in targeted radionuclide therapy for endocrine malignancies. *PET Clinics*.

[36] Evangelista L., Ravelli I., Bignotto A., Cecchin D., Zucchetta P. (2020). Ga-68 DOTA-peptides and F-18 FDG PET/CT in patients with neuroendocrine tumor: a review. *Clinical Imaging*.

[37] Gauthé M., Testart Dardel N., Ruiz Santiago F. (2018). Vertebral metastases from neuroendocrine tumours: how to avoid false positives on ^68^Ga-DOTA-TOC PET using CT pattern analysis?. *European Radiology*.

[38] Bastawrous S., Bhargava P., Behnia F., Djang D. S. W., Haseley D. R. (2014). Newer PET application with an old tracer: role of ^18^F-NaF skeletal PET/CT in oncologic practice. *RadioGraphics*.

[39] Zhu W., Cheng Y., Wang X. (2020). Head-to-head comparison of ^68^Ga-DOTA-JR11 and ^68^Ga-DOTATATE PET/CT in patients with metastatic, well-differentiated neuroendocrine tumors: a prospective study. *Journal of Nuclear Medicine*.

[40] Wang H., Du Z., Huang Q. (2021). The superiority of [^68^Ga]Ga-FAPI-04 over [^18^F]-FDG in a case of neuroendocrine tumour with hepatic metastasis. *European Journal of Nuclear Medicine and Molecular Imaging*.

[41] Cheng Z., Zou S., Cheng S., Song S., Zhu X. (2021). Comparison of ^18^F-FDG, ^68^Ga-FAPI, and ^68^Ga-DOTATATE PET/CT in a patient with pancreatic neuroendocrine tumor. *Clinical Nuclear Medicine*.

